# Soybean Trihelix Transcription Factors GmGT-2A and GmGT-2B Improve Plant Tolerance to Abiotic Stresses in Transgenic Arabidopsis

This article has been retracted.

**DOI:** 10.1371/journal.pone.0006898

**Published:** 2009-09-04

**Authors:** Zong-Ming Xie, Hong-Feng Zou, Gang Lei, Wei Wei, Qi-Yun Zhou, Can-Fang Niu, Yong Liao, Ai-Guo Tian, Biao Ma, Wan-Ke Zhang, Jin-Song Zhang, Shou-Yi Chen

**Affiliations:** 1 National Key Laboratory of Plant Genomics, Plant Gene Research Center, Institute of Genetics and Developmental Biology, Chinese Academy of Sciences, Beijing, China; 2 Graduate School of Chinese Academy of Sciences, Beijing, China; 3 Xinjiang Academy of Agricultural and Reclamation Science, Shihezi, China; Cairo University, Egypt

## Abstract

**Background:**

Trihelix transcription factors play important roles in light-regulated responses and other developmental processes. However, their functions in abiotic stress response are largely unclear. In this study, we identified two trihelix transcription factor genes *GmGT-2A* and *GmGT-2B* from soybean and further characterized their roles in abiotic stress tolerance.

**Findings:**

Both genes can be induced by various abiotic stresses, and the encoded proteins were localized in nuclear region. In yeast assay, GmGT-2B but not GmGT-2A exhibits ability of transcriptional activation and dimerization. The N-terminal peptide of 153 residues in GmGT-2B was the minimal activation domain and the middle region between the two trihelices mediated the dimerization of the GmGT-2B. Transactivation activity of the GmGT-2B was also confirmed in plant cells. DNA binding analysis using yeast one-hybrid assay revealed that GmGT-2A could bind to GT-1bx, GT-2bx, mGT-2bx-2 and D1 whereas GmGT-2B could bind to the latter three elements. Overexpression of the *GmGT-2A* and *GmGT-2B* improved plant tolerance to salt, freezing and drought stress in transgenic Arabidopsis plants. Moreover, *GmGT-2B*-transgenic plants had more green seedlings compared to Col-0 under ABA treatment. Many stress-responsive genes were altered in *GmGT-2A*- and *GmGT-2B-*transgenic plants.

**Conclusion:**

These results indicate that *GmGT-2A* and *GmGT-2B* confer stress tolerance through regulation of a common set of genes and specific sets of genes. GmGT-2B also affects ABA sensitivity.

## Introduction

Transcriptional regulation of gene expression plays a primary role in plant development and in environmental stimuli responses. Expressions of the stress-responsive effector genes are largely controlled by several classes of transcription factors, such as members of the MYB, ERF/AP2, bZIP, WRKY and NAC families, through binding of the corresponding *cis*-acting elements [1]–[7]. The potential for improving plant tolerance by engineering of stress-regulated transcription factors is highlighted recently [8].

Several classes of transcription factors such as AP2/ERF, DOF, YABBY and Trihelix families are unique to plant so far [9]–[14], suggesting that they may be implicated in plant-specific gene tuning [15]. Members of Trihelix family, also known as GT factors (DNA binding proteins with specificity for GT-elements), are among the first transcription factors identified in plants [16]. GT elements are highly degenerated and the deduced consensus core sequence is 5′-G-Pu-(T/A)-A-A-(T/A)-3′ [14], and are involved in a wide array of plant biological processes. GT elements were first identified in the pea rbcS-3A gene promoter as a light-responsive element named Box II/GT1 box (5′-GTGTGGTTAATATG-3′) [17], [18] and later in many promoters of other genes, some of which were not responsive for light [14]. For instance, a GT element named Site1, found in the ribosomal protein gene *rps1* promoter, has been shown to repress transcription in non-photosynthetic tissues or cells [19], [20]. Box II-related/GT-1 like elements found in the promoter region of soybean *chs* gene and *Pr-1A* gene from tobacco are likely responsive to elicitor treatments and pathogen infection [21], [22]. The pathogen- and NaCl- induced soybean *SCaM-4* gene contains GT-1 like element in the promoter region [23].

Rice GT-2 and tobacco GT1a/B2F were the first two nuclear proteins identified via affinity screening using GT2 sequence and Box II sequence [24]–[26]. Since then, more members of GT factor (trihelix transcriptional factor) family have been isolated from Arabidopsis, pea, soybean and rice [16], [27]–[32]. The trihelix transcriptional factor family has 28 members in Arabidopsis genome [33], 22 members in rice genome [34] and putatively 13 members in soybean genome [11], and is defined based on the highly conserved trihelix domain (helix-loop-helix-loop-helix). Members of trihelix family can be divided into three subgroups that bind to functionally distinct types of GT elements. GT-1-type factors contain only a single trihelix domain that is responsible for specific binding to the Box II core sequence, whereas GT-2-type factors contain twin trihelix domains with the N-terminal one preferentially binding to GT3-bx (5′-GAGGTAAATCCGCGA-3′) and the C-terminal one to GT2-bx(5′-GCGGTAATTAA-3′) [29], [30]. Although AtGT-3a and AtGT-3b are similar to GT-1 in structure that containing one single trihelix motif, both of them bind specifically to GT-3a site (core sequence 5′-GTTAC, i.e. Site 1), not to Box II, GT2-bx or GT3-bx *in vitro*, suggesting that they belong to a third subgroup of GT factors [27].

It is generally believed that trihelix factors are involved in the regulation of light-responsive genes [14], [35]. The expression of all of the trihelix factors cloned thus far appears to be ubiquitous and independent of light, except that *AtGTL1* mRNA is more abundant in siliques, and soybean *GmGT-2* and rice *rml1* (rice gene regulated by *Magnaporthe grisea* and light) were down-regulated by light [24]–[26], [29], [30], [32]. Arabidopsis *PETAL LOSS* (*PTL*) gene encoding a GT-2-type factor is the first member of trihelix family known to control morphogenesis [28]. A rice *Shattering 1*(*SHA1*) gene encoding a GT-1-type factor plays an important role in activation of cell separation, and a mutation in the trihelix domain resulted in the elimination of seed shattering in cultivated rice [31]. More recently, ASIL1, belonging to a new subfamily of the trihelix transcription factors, has been found to function as a negative regulator of a large subset of Arabidopsis embryonic and seed maturation genes in seedlings [36].

Although the roles of the trihelix factors are gradually disclosed, the regulatory function of this kind of transcription factors in abiotic stress response remains largely unknown. In a previous work, we have identified 13 putative trihelix genes in soybean [11]. From these, two abiotic stress-upregulated genes encoding putative GT-2-type proteins (named GmGT-2A and GmGT-2B, respectively) were cloned from soybean in this study. Both *GmGT-2A* and *GmGT-2B* overexpression in Arabidopsis plants increased plant tolerance to abiotic stresses. The downstream genes regulated by *GmGT-2A* and *GmGT-2B* were also investigated. GmGT-2A and GmGT-2B may represent the first two members of trihelix family that are responsible for the stress tolerance in transgenic Arabidopsis plants through regulation of downstream genes.

## Results

### Gene cloning and structural analysis of the trihelix family genes *GmGT-2A* and *GmGT-2B*

Among thirteen ESTs that belong to trihelix family genes from soybean, two were identified to be responsive to various abiotic stresses. The full-length coding regions of the two corresponding genes were further obtained using RACE method. Because both of them encoded proteins similar to those from the GT-2 group of the trihelix family [36], we named the two genes as *GmGT-2A* (EF221753) and *GmGT-2B* (EF221754) respectively and further analyzed.

SMART analysis revealed two trihelix domains in both the GmGT-2A and GmGT-2B proteins (Fig. 1A, C). Between these two trihelix domains, a coiled-coil region of 31 residues was noted in GmGT-2A. Four putative nuclear localization signals (NLS) were identified in GmGT-2A (Fig. 1C). However, only three NLSs were found in GmGT-2B and the second NLS appeared not present in this protein (Fig. 1C). It should be noted that an asparagine-rich region was found in the middle of the C-terminal trihelix domains of the GmGT-2A and GmGT-2B but not in other proteins compared (Fig. 1C). This feature possibly suggests a potentially specific function for this region in regulation of the transcription factor activity in soybean.

**Figure 1:** Schematic representation and amino acid sequence alignment of the GmGT-2A and GmGT-2B. (A) Schematic diagram of the GmGT-2A and GmGT-2B. (B) Cluster analysis of the GmGT-2A and GmGT-2B with other GT-2 group factors. The analysis was performed by using the MEGA 4.0 program with neighbor joining method and with 1000 replicates. Numbers on the figure are bootstrap values. The sequences are from soybean and Arabidopsis plants [36]. (C) Multiple alignments of the amino acid sequences from various GT factors. NLS indicates putative nuclear localization signal. Accession numbers are as follows: GmGT-2 (AF372498), GmGT-2A(EF221753), GmGT-2B(EF221754). Arabidopsis gene codes are as in [36].

The amino acid sequences of the GmGT-2A and GmGT-2B were compared with those from other homologous proteins (Fig. 1C). At the whole amino acid level, the GmGT-2A showed 39% identity with the GmGT-2 (O'Grady et al., 2001), but ∼25% identity with GmGT-2B and the other two proteins compared. GmGT-2B showed 22% identity with GmGT-2 and similar identity with other proteins. For the N- and C-terminal trihelix domains, GmGT-2A had 74% and 67% identity with those of GmGT-2, and 40% and 53% identity with those of GmGT-2B. GmGT-2B had 35% and 56% identity with those of GmGT-2. These results indicate that the GmGT-2A is more closely related to GmGT-2 but not the GmGT-2B. Cluster analysis also supports this conclusion (Fig. 1B). In addition, the soybean GmGT-2A, GmGT-2B and GmGT-2 are closely related to the GT-2 group of Arabidopsis but not clustered with other group members from Arabidopsis (Fig. 1B)[36].

### *GmGT-2A* and *GmGT-2B* gene expressions in different soybean organs and in response to abiotic stresses

The expressions of the *GmGT-2A* and *GmGT-2B* were examined in different organs of the soybean plants. The results in Figure 2A showed that the *GmGT-2A* was expressed in a higher level in stems than those in others organs tested, and no expression of this gene was detected in soybean seeds. For the *GmGT-2B*, its expression was higher in pods but lower in other organs examined. Similarly, the *GmGT-2B* showed no expression in soybean seeds.

**Figure 2:** Expressions of the *GmGT-2A* and *GmGT-2B*. (A) Gene expressions in different organs of soybean plants. RT-PCR method was used and tubulin gene was amplified as a control. (B) Expressions of the *GmGT-2A* and Gm*GT-2B* in response to ABA and stress treatments revealed by Northern analysis. *GmGT-2* expression was also compared. (C) Subcellular localization of the GmGT-2A and GmGT-2B as revealed by GFP fusion proteins. Green fluorescence indicates location of the GFP control or the GFP fusion proteins. Red fluorescence indicates positions of chloroplasts.

The soybean seedlings were treated with various stresses and the *GmGT-2A* and *GmGT-2B* gene expressions were investigated. Both gene expressions can be enhanced by ABA, cold, drought and salt treatments (Fig. 2B). However, the expression patterns were different. The *GmGT-2A* transcripts accumulated to a higher level at 12 h after initiation of the treatments with ABA, cold or drought stress, whereas the *GmGT-2B* expression had peak levels at 1 h and/or 3 h after the three treatments. The upregulation of *GmGT-2A* expression after 12-h ABA treatment may be an indirect effect. At 12 h after these treatments, the *GmGT-2B* expression was apparently declined (Fig. 2B). Under salt stress, the *GmGT-2A* and *GmGT-2B* inductions were similar in patterns. These results suggest that the *GmGT-2A* and *GmGT-2B* may be involved in regulation of plant responses to abiotic stresses. Because the *GT-2* gene showed similarity to the *GT-2A* and *GT-2B*, we further tested if this gene is responsive to stresses. However, after the four treatments, the *GT-2* expression was not significantly altered, indicating that the gene may not be involved in abiotic stress responses (Fig. 2B).

### Subcellular localization of the GmGT-2A and GmGT-2B

Because the GT-2A and GT-2B contained putative NLSs, we examined the subcellular localization of the two proteins. Each of the two genes was fused to the *GFP* and then transfected into Arabidopsis protoplasts to observe the localization of the GFP fusion proteins. The green fluorescence from GFP control was localized in both nuclear region and cytoplasm whereas the green fluorescence of the GmGT-2A-GFP and GmGT-2B-GFP fusion proteins was abundant in nuclear region of the protoplasts (Fig. 2C). The red fluorescence indicated the position of chloroplasts. These results indicate that the GmGT-2A and GmGT-2B are nuclear proteins.

### Transcriptional activation, dimerization and DNA binding analysis of the GmGT-2A and GmGT-2B

Because the GmGT-2A and GmGT-2B belong to the transcription factors of trihelix family, we studied the transcription activation ability of the two proteins using the yeast assay system (Fig. 3A). Constructs, which harbored various versions of GmGT-2A and GmGT-2B (Fig. 3B), were made in pBD vector and transfected into yeast strain YRG-2. The yeast transformants were examined for their growth on selection medium (SD-His) due to activation of the reporter *HIS3* gene, or determined for their β-galactosidase activity due to the activation of the reporter *LacZ* gene (Fig. 3A). Full-length of the GmGT-2A [GT-2A(FL)] did not had any transcriptional activation ability. Its N-terminal half [GT-2A(NT)] or C-terminal half [GT-2A(CT)] did not have the activity either (Fig. 3C). However, the full-length GmGT-2B had transcriptional activation activity, and its N-terminal half [GT-2B(NT)] also had the activity (Fig. 3C). The C-terminal half [GT-2B(CT)] did not had the transcriptional activation ability. The N-terminal half of the GmGT-2B was further truncated and the N-terminal peptide of 153 residues [GT-2B(N1-153)] were enough to have the activation ability. Further truncations including the GT-2B(N1-89), GT-2B-N_GT_(90-153) or the middle part of the GT-2B [GT-2B-M(150-424)] did not have any activation ability (Fig. 3C).

**Figure 3:** Transcriptional activation, dimerization and DNA binding analysis. (A) Schematic diagrams for transcriptional activation (left panel) and dimerization (right panel) in yeast assay. (B) Different versions of GmGT-2A and GmGT-2B used for the analysis. FL: full-length protein. NT: N-terminal region. CT: C-terminal region. Numbers indicate amino acid positions. (C) Transcriptional activation activity of different versions of the GmGT-2A and GmGT-2B. Growth of transformants on SD-His and blue color in the presence of X-Gal indicate that the corresponding proteins have transcriptional activation ability. (D) Dimerization analysis of GmGT-2A or GmGT-2B. Growth of the transformants on SD/-Trp-Leu-His plus 10 mM 3-AT (SD-3) and presence of blue color indicate positive interactions. Each version of proteins in pBD vector plus pAD vector, or each version in pAD vector plus pBD vector served as negative controls. (E) Identification of domains in GmGT-2B for dimerization. Others are as in (D). (F) DNA binding analysis. Growth of the transformants on SD/-Trp-Leu-His plus 3-AT indicates that the corresponding proteins can bind to the *cis*-DNA elements. D1: 5′-catctacagttactagctagt-3′; GT-1bx: 5′-gtgtggttaatatg-3′; GT-2bx: 5′-tggcggtaattaactg-3′; mGT-2bx-1: 5′-tggctttaattaactg-3′; mGT-2bx-2: 5′-tggcgggcattaactg-3′; mGT-2bx-3: 5′-tggcggtacgtaactg-3′; mGT-2bx-4: 5′-tggcggtaattgcctg-3′; CaM-4: 5′-gatccgcgtag-3′; GT-3b: 5′-taagaaaaataa-3′. (G) Transcriptional activation assay in Arabidopsis protoplasts. GALDBD is a negative control and VP16 is a positive control for transactivation ability. The GmGT-2B has transactiation activity whereas the GmGT-2A does not have the activity.

The dimerization ability of the two proteins was also analyzed and we find that the full-length protein of the GmGT-2B, the N-terminal half and the C-terminal half can form homodimers respectively (Fig. 3D). Other combinations did not produce any homo- or -herterodimers (Fig. 3D). Each version of proteins in pBD vector plus pAD vector, or each version in pAD vector plus pBD vector did not generate positive response (data not shown).

Because the GmGT-2B(NT) can form dimer, we then examined which part is responsible for the dimerization. Figure 3E showed that the middle part GT-2B-M(150–424) can form dimers whereas the N-terminal trihelix N_GT_ or C-terminal trihelix C_GT_ themselves can't form dimers. Other combinations did not generate dimerizations.

DNA-binding ability was investigated using yeast one-hybrid system. The effector plasmids harboring the GmGT-2A, GmGT-2B or their truncated forms were made in pAD vector, and the reporter plasmid was made by inserting four tandem repeats of various *cis*-DNA elements into the pHIS2, which contained a reporter gene *HIS3*. A minimal promoter was present downstream of the tested *cis*-DNA elements but upstream from the *HIS3* gene. The effector plasmids and the reporter plasmids were transfected into yeast strain Y187 and growth of the transformants on SD/-Trp-Leu-His plus 3-AT indicates binding of the transcription factors to the corresponding *cis*-DNA elements. Figure 3F showed that the GmGT-2A, GmGT-2B, and their N-terminal or C-terminal truncated versions all can bind to the GT-2bx, the mGT-2bx-2, and the D1 element. However, the C-terminal region of GmGT-2A or GmGT-2B appeared to have low affinity for the D1 element. In addition, the GmGT-2A, its N-terminal and C-terminal region can bind to the GT-1bx (Fig. 3F). The GmGT-2A, GmGT-2B or their truncated versions could not bind to other elements tested. These results indicate that the GmGT-2A and GmGT-2B had common features in DNA binding and the GmGT-2A also had specialty in this ability.

The transcriptional activation ability was further examined in Arabidopsis protoplast assay system. Effector plasmids containing the *GmGT-2A* or *GmGT-2B*, and a reporter plasmid containing a firefly luciferase (LUC) gene were co-transfected into Arabidopsis protoplasts and the relative LUC activity was determined. Figure 3G showed that the GmGT-2B protein activated higher level of reporter LUC activity than the negative control GALDBD. However, the GmGT-2A did not promote the reporter LUC activity. These results indicate that the GmGT-2B has transcriptional activation ability in the protoplast assay whereas the GmGT-2A does not have this ability.

### Seedling growth of the transgenic Arabidopsis plants overexpressing the *GmGT-2A* or *GmGT-2B* under ABA and osmotic stress

To investigate the biological function of the *GmGT-2A* and *GmGT-2B* gene in plant, we transformed the two genes driven by the 35S promoter into Arabidopsis plants and homozygous transgenic lines with higher gene expressions were used for further analysis (Fig. 4A). Throughout the plant growth and developmental stages, no significant difference was observed for these transgenic lines in comparison with the wild type plants grown under normal condition.

**Figure 4:** Morphogenesis of *GmGT-2A*- and *GmGT-2B*-transgenic seedlings under ABA and mannitol treatment. (A) Transgene expression in various transgenic lines as revealed by Northern analysis. (B) Seedling morphogenesis under ABA and mannitol treatment. (C) Green seedling rate in response to ABA. (D) Green seedling rate under mannitol treatment. For (C) and (D), each data point is average of three experiments (n = 150 for each experiment) and bars indicate SD. Asterisks indicate highly significant difference (P<0.01) from Col-0.

Because the *GmGT-2A* and *GmGT-2B* expressions were upregulated by ABA and various abiotic stresses (Fig. 2B), we examined the effects of ABA and stress treatment on seed germination and seedling growth of the transgenic plants. Seed germination was not significantly affected by the ABA, mannitol and salt treatments when compared with the wild type plants (data not shown). However, the morphogenesis of seedlings was altered. Under treatments with both 0.5 µM and 0.75 µM ABA, the *GmGT-2B*-transgenic lines (L11 and L69) exhibited significantly higher green seedling rates (∼30% to ∼40%) when compared with the rates in wild type plants (∼9% to ∼16%) (Fig. 4B, C). Under the same ABA treatments, the *GmGT-2A*-transgenic lines (L19 and L27) did not show significant change in the green seedling rate in comparison with that in the wild type plants. These results indicate that the *GmGT-2B* can promote seedling morphogenesis in the presence of ABA, possibly through suppression of ABA function. The transgenic seeds were also germinated on medium with mannitol and the green seedling rates were not significantly changed in the *GmGT-2A-* and *GmGT-2B*-transgenic plants (∼70% to ∼77%) in comparison with the rate in wild type plants (71%) (Fig. 4B, D). These results indicate that overexpression of the *GmGT-2B* conferred reduced sensitivity to ABA in the transgenic plants.

### Effects of salt stress on the transgenic plants overexpressing the *GmGT-2A* or *GmGT-2B*

Performance of the *GmGT-2A-*, *GmGT-2B*-transgenic plants under NaCl treatment was examined. Under normal condition, all the transgenic lines showed no significant difference when compared with the wild type plants in terms of the phenotype and the survival rate (Fig. 5A, B). Treatments with 75 mM or 125mM NaCl did not affect the survival of all the transgenic lines compared either (Fig. 5A; data not shown). Under 150 mM NaCl treatment, ∼12% of the wild type plants were dead whereas all the *GmGT-2A*- and *GmGT-2B*-transgenic plants survived (Fig. 5A, B). The survival rate was further reduced at the 180 mM NaCl treatment, with the wild type plants having a survival rate of around 70%. On the contrary, the *GmGT-2A*- and *GmGT-2B*-transgenic plants had a survival rate of more than 90% (Fig. 5A, B).

**Figure 5:** Performance of the *GmGT-2A*- and *GmGT-2B*-transgenic plants under salt stress. (A) Growth of the transgenic seedlings in NaCl medium. (B) Survival rate of the salt-treated plants in (A). (C) Comparison of growth of the salt-treated plants in pots. Plants from treatments as in (A) were transferred in pots and the pictures were taken at 8 d and 21 d after transfer. (D) Survival rate of the salt-treated plants in pots from (C). For (B) and (D), each data point is average of three experiments (n = 30 for each experiment) and bars indicate SD. Asterisks indicate highly significant difference (P<0.01) from Col-0.

The salt-stressed seedlings on plates (Fig. 5A) were further transferred in pots containing vermiculite and their recovery at 8 d and 21 d was observed. Treatments with 75 mM and 125 mM NaCl did not significantly affect recovery of all the compared plants (Fig. 5C). However, at 150 mM NaCl, the recovery rate was reduced to ∼50% for the wild type plants whereas this rate was more than 80% for all the transgenic lines. At 180 mM NaCl, the recovery for the wild type plants was ∼25%. For both the *GmGT-2A*- and *GmGT-2B*-transgenic plants, the recovery rates were more than 90% (Fig. 5C, D). All these results indicate that the GmGT-2A and GmGT-2B conferred plant tolerance to salt stress.

### The *GmGT-2A* and *GmGT-2B* confer drought and freezing tolerance in their transgenic Arabidopsis plants

Because expression of the *GmGT-2A* and *GmGT-2B* genes can be induced under drought and cold treatments, we investigated if the performance of their transgenic plants was altered under these stresses. Plants (12-day-old) in pots were subjected to drought stress by withholding water for 16 d. After this stress, only ∼40% of the wild type plants survived whereas more than 90% of the *GmGT-2A*- and *GmGT-2B*-transgenic plants can survive and grow well (Fig. 6A, B). All the plants under normal condition grew normally (Fig. 6A). Plants that start to have siliques were further treated under drought stress by withholding water from plants for 16 d. The aerial parts of these plants were harvested and the dry weights of the transgenic plants were significantly higher than that of the wild type plants (Fig. 6C). These results indicate that the GmGT-2A and GmGT-2B confer drought tolerance to the transgenic plants.

**Figure 6:** Performance of the *GmGT-2A*- and *GmGT-2B*-transgenic plants under drought and freezing stress. (A) Phenotype of the transgenic plants under drought stress. (B) Survival rate of the transgenic plants under drought stress. Each data point is average of three experiments (n = 30 for each experiment) and bars indicate SD. (C) Comparison of plant dry weight after drought stress. Bars indicate SD (n = 30). (D) Water loss in detached leaves from the transgenic plants. Bars indicate SD (n = 3). (E) Water contents in aerial part of the pot-grown plants after withholding water. Bars indicate SD (n = 8). (F) Survival of the transgenic plants under freezing treatment after aclimation or non-acclimation. (G) Survival rate of the transgenic plants after treatment in (F). Each data point is average of three experiments (n = 30 for each experiment) and bars indicate SD. For (B), (C), (E), (G), asterisks indicate a significant difference (*P<0.05 and ** P<0.01) from Col-0.

Water loss represents another parameter for estimation of the plant tolerance to drought stress. Transgenic plants overexpressing the *GmGT-2A* or *GmGT-2B* all had reduced water loss in comparison with the wild type plants when detached leaves were used for the desiccation analysis (Fig. 6D). The whole plants (six-week-old) were also withheld from water for various times and the aerial parts were measured for water content. Figure 6E showed that, at day 8 and day 12 after the treatment, the water content was significantly higher in one *GmGT-2A*-transgenic line and two *GmGT-2B*-transgenic lines compared to the control plants, suggesting that these transgenic plants are tolerant to drought stress.

Nonacclimated or cold-acclimated (5 d at 4°C) 12-day-old seedlings were exposed to freezing temperature for 6 h and then the plants were returned to normal conditions for evaluation of performance after 7-d recovery. All the transgenic lines showed a better growth than the WT control, and the acclimated transgenic plants had higher survival rate after freezing treatment at different temperatures when compared to the nonacclimated transgenic plants (Fig. 6F, G). Under normal condition, all the plants grew very well (Fig. 6F). In addition, the *GmGT-2B*-overexpressing plants had a higher survival rate than the *GmGT-2A*-overexpressing plants under both acclimated and nonacclimated condition (Fig. 6G). These results indicate that overexpression of both the *GmGT-2A* and *GmGT-2B* improved plant tolerance to freezing.

### GmGT-2A and GmGT-2B regulate expressions of stress-responsive genes

The GmGT-2A and GmGT-2B may function in plant stress tolerance through regulation of downstream genes. We selected 33 stress-responsive genes for further quantitative real-time PCR analysis. Figure 7 showed that 17 genes including *AZF1, MYB74, MYB75, PAD3, LTP3, STZ, MYB73, LTP4, At4g30650, UGT71B6, RHL41, COR13, MYB77, CYP707A3, LTI30, RCI3*, and *DREB2A* were enhanced in all the transgenic lines harboring the *GmGT-2A* or *GmGT-2B*. The *AZF1*, *STZ* and *RHL41/Zat12* encoded plant-specific transcription factors with Cys-2/His-2 zinc finger motifs, and can be induced by various stresses. Overexpression of the STZ, Zat10 and Zat12 increased stress tolerance [37]–[39]. The four MYB genes *MYB73, MYB74, MYB75* and *MYB77* can be induced by salt stress [40], [41]. The *LTP3, LTP4, PAD3* and UGT71B6 were involved in ABA responses [42]–[44]. The At4g30650, *COR13* and *LTI30* were also involved in abiotic stress response [45], [46]. *CYP707A3* encodes an ABA 8′-hydroxylase. The *cyp707a3* mutant plants are hypersensitive to ABA and exhibited enhanced drought tolerance [47]. *RCI3* encodes a peroxidase and overexpression of the gene conferred dehydration and salt tolerance [48]. DREB2A expression does not activate downstream genes under normal growth condition. However, overexpression of its constitutive active form leads to drought stress tolerance and slight freezing tolerance [49].

**Figure 7:** Altered gene expressions in *GmGT-2A*- and *GmGT-2B*-transgenic plants in comparison with the WT (Col-0). For each gene, two transgenic lines were used. The quantitative RT-PCR was used for the analysis. Totally 33 genes were examined for their expressions. Bars indicate SD (n = 4).

Two genes *MYB90* and At4g02200 were only highly expressed in the *GmGT-2A*-transgenic plants compared to the control and the *GmGT-2B*-transgenic plants. Eleven genes including *MYB47, MYB15, PAD3, LTP3, LTP4, CBF2, PMZ, COR13, HVA22E, CBF1*, and *NCED3* were highly expressed in *GmGT-2B*-transgenic plants compared to the control plants and *GmGT-2A*-transgenic plants. These genes have been found to be responsive to various abiotic stresses and/or ABA response [41], [42], [50], [51]. The *NCED* genes have been found to be responsible for the biosynthesis of ABA precursor and are also involved in regulation of plant responses to abiotic stresses [52], [53]. Six genes including *LHY1, MYB2, At5g02840, VAMP711, At3g09600*, and *CCA1* were downregulated in all the transgenic lines. The *LHY1, CCA1, At5g02840* and *MYB2* have been found to be responsive to stress and/or ABA [41], [54]. Transgenic plants overexpressing *MYB2* had higher sensitivity to ABA and showed stress tolerance [55]. Suppression of the *VAMP711*, a gene encoding a protein for vesicle trafficking, in antisense transgenic plants improved salt tolerance [56].The gene *PK1/PK6*, which was induced by different stresses [57], was inhibited in the *GmGT-2A*-transgenic lines but promoted in the *GmGT-2B*-transgenic lines. These results indicate that *GmGT-2A* and *GmGT-2B* regulated a common set of genes as well as specific sets of genes for stress tolerance.

## Discussion

Although roles of trihelix family transcription factors have been discovered in light-relevant and other developmental processes, their functions in abiotic stress response are largely unknown. In the present study, two trihelix family transcription factor genes *GmGT-2A* and *GmGT-2B* from soybean were identified to be stress-responsive and conferred stress-tolerance in transgenic Arabidopsis plants through regulation of downstream genes. This study adds the trihelix family members to those transcription factors that can improve plant stress-tolerance.

The GmGT-2B exhibited transcriptional activation activity in both the yeast assay and the protoplast assay, whereas the GmGT-2A did not have this activity. This difference in transcriptional activation ability may result in the differential gene expressions in the transgenic plants, with more genes being highly or specifically expressed in the *GmGT-2B*-transgenic plants (Fig. 7). The activation domain of the GmGT-2B was also analyzed in detail and it appears that the N-terminal peptide of 153 residues is the minimal domain for transcriptional activation. Neither the N-terminal trihelix domain (90–153) nor its N-terminal sequence (1–89) themselves has the ability to activate transcription. The role of the minimal activation domain needs to be further tested in plant system. A rice GT-2 protein has also been found to function as a transcriptional activator. However, the activation domain was not identified [58]. Arabidopsis GT-1 also has transactivation function in both yeast and plant cells [59]. However, ASIL1 functions as a repressor for embryonic and seed maturation genes in Arabidopis seedlings [36]. The present GmGT-2A does not have transcriptional activation ability (Fig. 3C, G). Whether it has repression activity needs further study.

The GmGT-2B, unlike the GmGT-2A, has the ability to dimerize, and the dimerization seems to happen through interaction of the middle part of the protein. No heterodimers could be formed between GmGT-2A and GmGT-2B. The biological significance of such interaction is not known. It is possible that the interaction would modify the transcriptional activation ability and then affect the downstream gene expressions. Arabidopsis GT-3a and GT-3b could form homo or heterodimers, and the dimerization domain seemed to be located at the C-terminus. However, no interaction was observed between each of the two proteins with the GT-1 [27].

The trihelix domain is generally believed to be the DNA-binding domain [29], [30]. In the yeast one-hybrid assay, both the N-terminal and C-terminal trihelix-domain-containing region of the GmGT-2A and GmGT-2B can bind to the three elements (Fig. 3F). In addition, the GmGT-2A can bind to the GT-1 bx whereas the GmGT-2B can't. These different features imply that the two genes may play some different roles in plant. However, since the two genes also have common features in gene expression and DNA-binding, they should also have similar functions in addition to their specific functions.

Seed germination and seedling morphogenesis can be inhibited by ABA (Fig. 4). The germination rates of the *GmGT-2A*- and *GmGT-2B*-transgenic seeds were similar to that of the wild type seeds with ABA treatment (data not shown), indicating that the two genes did not affect ABA-regulated germination process. It is interesting to find that the morphogenesis of the *GmGT-2B*-transgenic seedlings but not the *GmGT-2A*-transgenic seedlings was less affected by ABA treatment. This fact suggests that the *GmGT-2B*-transgenic plants have reduced sensitivity to ABA, and *GmGT-2B* may function as a negative regulator to suppress the ABA effects on morphogenesis. Downstream gene analysis revealed that a number of genes had much higher expression in the *GmGT-2B*-transgenic plants than that in the *GmGT-2A*-transgenic plants (Fig. 7), and these genes may contribute to the reduced ABA sensitivity in the *GmGT-2B*-transgenic plants. Alternatively, these *GmGT-2B*-upregulated genes may reflect a positive feedback of the ABA response due to the reduction of ABA sensitivity. In fact, several ABA-regulated or related genes including *NCED3, LTP3, LTP4* and *PAD3* etc. were enhanced in the *GmGT-2B*-transgenic plants. These studies on ABA effects may also suggest that *GmGT-2B* plays larger roles than *GmGT-2A* in regulation of seedling morphogenesis.

The *GmGT-2A* and *GmGT-2B* showed differential expression in response to ABA and other stresses. However, expression of their homologue *GmGT-2* was not induced by these treatments, suggesting that the *GmGT-2A* and *GmGT-2B* have specific roles in abiotic stress responses. Overexpression of both the *GmGT-2A* and *GmGT-2B* greatly improved plant tolerance to salt, freezing and drought stresses as can be seen from the survival rates of the transgenic plants, the dry weight and the water loss (Fig. 5, 6). The regulation of stress tolerance may be achieved through control at levels of transcriptional activation, DNA binding, and dimerization and/or by other unknown mechanisms. These controls at different levels will finally affect gene expressions, through which the stress tolerance can be achieved in plants. Actually, many genes have been found to be upregulated in the transgenic plants. Among these, three C2/H2 zinc finger-type transcription factors were increased and may play significant roles since two of the genes *STZ* and *RHL41/Zat12* have been found to promote stress tolerance [37], [38], [51]. *DREB2A* gene and a peroxidase gene *RCI3* were also highly expressed in the *GmGT-2A*- and *GmGT-2B*-transgenic plants. These two genes have been found to improve stress tolerance in transgenic plants [48], [49]. Therefore, the GmGT-2A and GmGT-2B may at least activate these gene expressions either through direct binding to promoter of each gene or in a manner of indirect regulation. Expression of a few genes were also suppressed by the two *GmGT* genes. The *VAMP711*, a gene encoding a protein related to vesicle trafficking, was downregulated. Suppression of the *VAMP711* inhibited the fusion of the H_2_O_2_-containing vesicle to the tonoplast, leading to improved vacuolar functions for plant salt tolerance [56]. It is therefore possible that the present two GmGT genes conferred stress tolerance at least through activation of STZ/ZAT and DREB2A transcription factors as well as the antioxidative system. Moreover, the *GmGT-2B*-transgenic plants appeared to be slightly more tolerant to stresses than the *GmGT-2A*-transgenic plants did (Fig. 5B, 6G). This difference is most likely due to the higher expressions of the specific genes in *GmGT-2B*-transgenic plants (Fig. 7). It should be mentioned that overexpression of the transcription factors in Arabidopsis plants might induce tolerance observations not related to activation of specific pathways but rather indirect or pleiotropic effects. Further transgenic analysis in soybean plants may disclose such a possibility.

Overexpression of the *GmGT-2B* gene resulted in reduced ABA sensitivity (Fig. 4), but still improved plant tolerance to salt, drought and freezing stress (Fig. 5, 6). This phenomenon appears to be inconsistent with the notion that ABA insensitivity would generally lead to reduced stress tolerance. However, our results were in line with several reports showing that genes conferring reduced ABA sensitivity can increase stress tolerance. Yang et al. [60] found that Lily hydrophilin gene *LLA23*-transgenic seeds showed reduced sensitivity to ABA, however, its transgenic plants exhibited tolerance to salt, osmotic and drought stresses. An ABF2-interacting protein gene *ARIA*-overexpressing plants are hypersensitive to ABA but also sensitive to high osmolarity during germination [61]. Transgenic plants overexpressing *GmbZIP44*, *GmbZIP62* and *GmbZIP78* from soybean show reduced sensitivity to ABA but enhanced tolerance to salt and freezing stress [5].

It should be mentioned that the GmGT-2A does not have transcriptional activation activity and could not form homo or heterodimers. However, it still can bind to *cis*-DNA elements and improve stress tolerance through alteration of gene expressions. The GmGT-2A may need post-translational modification to achieve its transcriptional activation. Other mechanisms may also be involved.

Overall, we have identified two GT factors GmGT-2A and GmGT-2B from soybean, whose overexpression differentially regulated seedling morphogenesis and improved plant tolerance to abiotic stresses. The stress tolerance conferred by these two factors is achieved by upregulation of a number of downstream genes. Further study should disclose more about the mechanism through which the two GT factors regulate plant stress responses.

## Materials and Methods

### Plant growth

Seeds of soybean (Glycin max, Nannong 1138-2) were grown in pots at 25°C under continuous light. Seedlings of 15-day-old were carefully pulled out from the vermiculite, rinsed and subjected to various treatments. For salt treatment, seedlings were immersed with the roots in 150 mM NaCl. For drought stress, seedlings were placed on filter papers at room temperature for air drying. For cold treatment, seedlings were placed in a beaker containing 4°C water. For ABA treatment, seedlings were immersed with the roots in 100 µM ABA. Seedlings were also placed in water at room temperature as a control treatment. After treated for the indicated times, the materials were harvested for RNA isolation. Roots, stems, leaves and cotyledons from 15-day-old seedlings, and flowers, young pods, and seeds from mature plants were also collected for examination of gene expression.

### Gene cloning

Two ESTs representing the middle parts of two trihelix family genes were found to be inducible under various abiotic stresses. 5′- and 3′-RACE were performed to obtain the full-length of the two genes. Finally the two genes were cloned into the pMD18-T vector to generate the original plasmids pMD18-T-GmGT-2A and pMD18-T-GmGT-2B for further use. The coding sequences of the two genes have been deposited into the GenBank under the accession numbers of EF221753 for *GmGT-2A* and EF221754 for *GmGT-2B*.

### Northern hybridization and RT-PCR analysis

Total RNA isolation and Northern hybridization followed previous descriptions by Zhang et al.[62]. Gene expressions were also examined by RT-PCR. For GmGT-2A, primers are 5′-AGGAAACCCCGCTAGAGAAC-3′ and 5′-GTTGTTGTCGGTTGTTGTCG-3′. For GmGT-2B, primers are 5′- GTTTTTGCGAGAGCATTGTG-3′ and 5′-AACTAGGGTTCTGGGGAGGA-3′. For GmGT-2, primers are 5′-GATTCCAAGACTTGTCCCTA-3′ and 5′-CCTATCACATTTCACTCCC-3′. Primers used for gene expressions in the transgenic Arabidopsis plants are listed in File S1.

### Transcriptional activation and dimerization analysis

Transcriptional activation analysis was based on previous method [12]. The full-length of the coding region of the *GmGT-2A* or *GmGT-2B* gene was cloned into the pBD vector to generate the pBD-GmGT-2A(FL) or pBD-GmGT-2B(FL). The N-terminal region containing N-terminal trihelix domain plus the sequence between the two trihelix domains was also cloned into the same vector to generate pBD-GmGT-2A(NT) or pBD-GmGT-2B(NT). Similarly, the C-terminal region containing the sequence between the two trihelix domains plus the C-terminal trihelix domain was cloned to generate pBD-GmGT-2A(CT) or pBD-GmGT-2B(CT). The N-terminal region of the GmGT-2B was further truncated and pBD-GmGT-2B(N1-89), pBD-GmGT-2B(N1-153) and pBD-GmGT-2B-N_GT_(90-153) were made. Further more, the C-terminal trihelix domain and the sequence between the two trihelix domains were used to construct pBD-GmGT-2B-C_GT_(425–492) and pBD-GmGT-2B-M(150–424) respectively. All the primers used for the transcriptional activation analysis are listed in File S1. BD vector and pBD-GAL4 were used as negative and positive controls respectively. Each plasmid was transfected into the yeast strain YRG-2 containing the *HIS3* and *LacZ* reporter genes. The transfected cells were examined for their growth on SD/-His or for the activity of β-galactosidase.

For dimerization analysis, the above full-length genes or truncated versions were also inserted into pAD vector to generate pAD-GmGT-2A/2B(FL), pAD-GmGT-2A/2B(NT), or pAD-GmGT-2A/2B(CT). For GmGT-2B, pAD-GmGT-2B-N_GT_(90–153), pAD-GmGT-2B-C_GT_(425–492) and pAD-GmGT-2B-M(150–424) were also constructed. The pBD-GmGT-2A/2B and pAD-GmGT-2A/2B were co-transfected into YGR-2 cells, and the transfected cells were observed for growth on SD/-Trp-Leu-His plus 10 mM 3-AT as previously described [63]. The activity of β-galactosidase was also examined.

### Transcriptional activation assay in *Arabidopsis* protoplasts

Full length sequences of *GmGT-2A* and *GmGT-2B* were obtained by PCR with the same primers as used in followed localization experiments. The GAL4 DNA-binding domain (BD)-coding sequence was fused to the above two genes and inserted into the pRT107 to generate effector plasmids pRT-BD-GmGTs. The fusion genes were under the control of 35S promoter. The BD sequence was also fused to VP16 gene to generate positive control effector plasmid. The pRT107 containing the BD sequence was used as negative control. The reporter plasmid containing 5X UAS and 35S promoter upstream of a reporter gene encoding a firefly luciferase (LUC) was used. The effector and reporter plasmids were co-transfected into Arabidopsis protoplasts and the relative LUC activity was determined based on previous descriptions [5]. The experiments have been repeated independently for three times and the results were consistent. Results from one experiment were presented.

### DNA binding analysis using yeast one-hybrid assay

The yeast one-hybrid assay followed previous description [12]. Four copies of each of the *cis*-DNA element, with SacI and MluI adaptors, were synthesized, annealed and cloned into the reporter plasmid pHIS2, which contains the reporter gene *HIS3*. Each of the pAD-GmGT-2A/2B(FL), pAD-GmGT-2A/2B(NT), or pAD-GmGT-2A/2B(CT) was co-transfected with each pHIS2 plasmid harboring different *cis*-DNA elements into the yeast cells (Y187). The transfected cells were examined for their growth on SD/-Trp-Leu-His plus 30 mM 3-AT.

### Localization of the GmGT in *Arabidopsis* protoplasts and confocal microscopic analysis

The full length sequence of *GmGT-2A and GmGT-2B* were cloned into the GFP221 plasmid to construct fusion plasmids using specific primers containing B*am*HI and *Sal*I sites. Primers 5′-CGCGGATCCATGCTGGAAATCTCAACT-3′ and 5′-ACGCGTCGACACTCATAATTGCAATGGA-3′ for Gm-GT-2A, 5′-CGCGGATCCATGTTCGATGGAGTACCA-3′ and 5′-ACGCGTCGACAAACTGATCAAAATCCAA-3′ for Gm-GT-2B were used. GFP221 plasmid containing a 35S-driven *GFP* gene was used as a control. The fusion construct or control plasmid was then introduced into *Arabidopsis* protoplasts (http://genetics.mgh.harvard.edu/sheenweb/protocols/) for confocal analysis using a Leica TCS SP5 microscope.

### Generation of transgenic Arabidopsis plants

The coding region of the *GmGT-2A* and *GmGT-2B* was amplified from their original plasmids with primers containing BamHI/SacI sites, and cloned into the pBI121 vector. The two genes were driven by the 35S promoter. For *GmGT-2A*, primers were 5′-gtcggatcc atgctggaaatctcaacttc-3′ and 5′-cgagagctcttaactcataattgcaatgg-3′. For GmGT-2B, primers were 5′-aacggatccatgttcgatggagtaccagacc-3′ and 5′-atcgagctcttaaaactgatcaaaatccaaag-3. The expression plasmids pBI-GmGT-2A/2B were transfected into agrobacterium GV3101 and then transformed into Arabidopsis plants using floral dip method. T3 homozygous plants with higher transgene expression were used for further analysis.

### Evaluation of stress tolerance for the transgenic Arabidopsis plants

Seeds from Arabidopsis thaliana Columbia (Col-0) ecotype or various transgenic lines were sown on Murashige and Skoog medium, stratified at 4°C for 3 d and incubated at 22°C under continuous light. Seedlings were transferred to plates containing ABA or mannitol to observe their effects on seedling morphogenesis after growth for 16 d. For NaCl treatment, 7-day-old seedlings were transferred onto medium containing different concentrations of NaCl and maintained for 16 d. These plants were further transferred into pots containing vermiculite and grown under normal condition for 8 d and 21 d. The pictures were taken and the survival rates of these plants were evaluated at different periods.

Freezing treatments were carried out according to Cuevas's method [64]. The tests were carried out in a temperature programmable freezer. Nonacclimated or cold-acclimated (5 d, 4°C) 12-day-old seedlings were exposed to 4°C for 30 min in darkness and subsequently the temperature was lowered at a rate of 2°C per hour. The final desired freezing temperature was maintained for 6 h, and then the temperature was increased again to 4°C at the same rate. After thawing at 4°C for 4 h in the dark, plants were returned to normal conditions. Tolerance to freezing was determined as the capacity of plants to resume growth after 7 d of recovery under control conditions.

For drought treatment, 12-day-old seedlings in pots were withheld from water for 16 d at 28°C with relative humidity of 20%. Plants at silique stage were also withheld from water for 16 d and the dry weight was measured and compared. Equal amount of vermiculite was added to each pot for comparison of plant growth and stress response.

For water loss measurements, leaves were detached from plants at the rosette stage and weighed immediately on a weighing paper. The weight was measured at designated time intervals. There were three replicates for each transgenic line. The percentage loss of fresh weight was calculated based on the initial weight of the plants [5].

Water content was measured according to previous descriptions with modifications [65]. Six-week-old plants in pots were withheld from water for 3 d, and then measurements were made every 4 d and lasted for 12 d. Aerial parts of eight plants were excised and fresh weight was measured. The materials were dried in an oven at 37°C for 4 d until constant weight. The relative water content was calculated.

### qRT-PCR analysis

Total RNA from aerial parts of four-week-old plate-grown plants was used for reverse-transcription (RT) with MMLV reverse transcriptase according to the manufacture's protocol (Promega). Genes selected and corresponding primers were shown in File S1. Real-time PCR were performed on MJ PTC-200 Peltier Thermal Cycler based on previous descriptions [5]. The real-time PCR results were analyzed using Opticon Monitor™ analysis software 3.1 (Bio-Rad).

### Statistical analysis

The data were subjected to statistic analysis, and analysis of variance was performed using the SPSS 12.0 program.

## Supporting Information

File S1 Primers used for transcriptional activation analysis and qRT-PCR analysis
(0.10 MB DOC)
